# Algorithm Composition and Emotion Recognition Based on Machine Learning

**DOI:** 10.1155/2022/1092383

**Published:** 2022-06-06

**Authors:** Jiao He

**Affiliations:** Wuhan Sports University, Wuhan 430079, China

## Abstract

This paper proposes a new algorithm composition network from the perspective of machine learning, based on an in-depth study of related literature. At the same time, this paper examines the characteristics of music and develops a model for recognising musical emotions. Using the model's information entropy of pitch and intensity to extract the main melody track, note features are extracted from bar features. Finally, the cosine of the vector included angle is used to judge the similarity between feature vectors of several adjacent sections, allowing the music to be divided into several independent segments. The emotional model of music is used to analyze each segment's emotion. By quantifying music features, this paper classifies and quantifies music emotion based on the mapping relationship between music features and emotion. Music emotion can be accurately identified by the model. The model's emotion recognition accuracy is up to 93.78 percent, and the algorithm's recall rate is up to 96.3 percent, according to simulation results. The recognition method used in this paper has a higher recognition ability than other methods, and the emotion recognition result is more reliable. This paper can not only meet the composer's auxiliary creative needs, but it can also help intelligent music services.

## 1. Introduction

With the development of economy and society, people put forward higher requirements for spiritual life. In today's society, people's entertainment life is richer and more diverse, and music is a special social ideology, which can not only cultivate sentiment and regulate emotions, but also develop thinking and glow emotions, and it has a strong appeal [1]. Music is becoming increasingly important in human life as a spiritual food. Simultaneously, digitalization, as the core of information technology, has aided the rapid development of a variety of emerging technologies; digitalization of audio has become the digital trend's intermediate force. As a result, the marriage of computer and music has become a research hotspot [2]. “Computer music” is a new technology that combines music art and computer technology. It is an important component of multimedia technology. Music has a higher scientific and technological content, as well as its own distinct and colourful artistic expression. The use of algorithms to create musical works is known as computer composition. One method of composing music is to use an algorithm set [3]. More researchers have devoted themselves to the research field of algorithmic composition because concrete music and random music differ greatly from the theoretical system and creative thinking of traditional composition techniques. Probability model, rule system model, genetic algorithm model, and NN (neural network) model are the most commonly used algorithm composing methods today. The motivation of composition and the development of motivation are precisely the application of these thoughts as the guidance of technological innovation in the universal law of music creation. The composition algorithm is both a simple mathematical operation and an expression of the artistry that exists in human thought. Computer automatic composition will greatly improve music creativity as machine learning advances, while also assisting composers in generating new creative ideas. However, as the amount of music produced grows, it is becoming increasingly important to classify and manage it.

The application of algorithms to solve specific problems is at the heart of algorithmic composition on a theoretical level, and the knowledge contained therein comes from musicology, mathematics, computer science, and other disciplines. These levels encompass not only specific technical methods of theoretical techniques and mathematical operations, but also a deeper expression of human thought. Music comes from life and reflects the creators' emotions [4]. Music is a psychological process that includes a variety of human emotional factors that are produced when people interact with music. Because of its heavy workload, difficult description, and impersonality, the early text annotation method has some limitations. Furthermore, as digital music production technology advances and the number of different types of music styles grows, text-based music retrieval becomes obsolete, and people begin to investigate new classification retrieval methods to aid in the retrieval of target music from massive data. The advantages of digital music over traditional music are primarily in the areas of production, storage, dissemination, and retrieval. Users' demand for music emotion can be met by emotion-based retrieval. In addition, a real-time soundtrack for multimedia video should be created based on the emotion conveyed by the video content. Music emotion recognition is a pattern recognition task, and the mapping of data from high-dimensional music feature space to low-dimensional emotion space must be done correctly. However, most musical emotion studies are limited to categorising an entire piece of music into one emotional category. Music's emotion, on the other hand, is not static. This paper uses a machine learning algorithm to create a model of music composition and emotion recognition. The following are some of its innovations:

1. There is basically no complete set of music data expression rules in algorithmic composition system. Based on the in-depth study of related literature, this paper proposes a new algorithm composition network from the perspective of machine learning algorithm [5–7]. It restrains the style and quality of generated music by using music theory rules to construct a reasonable Reward function. At the same time, the general machine learning methods created by deep learning network in the field of algorithm are summarized, so as to generate music with polyphonic structure. It can meet the composer's auxiliary creative needs and provide more support for intelligent music services.
2. In this paper, the average pitch, average sound intensity, speed, and other characteristics are analyzed, and the classification model of emotion feature vector input is constructed. It can select an appropriate formula according to the applied scene; at the same time, several adjustable parameters are set to adjust the similarity. This paper classifies and quantifies music emotion according to the mapping relationship between music characteristics and emotion by quantifying music characteristics. The model can accurately identify the emotion of music.

## 2. Related Work

Computer-aided music creation and algorithm-based music creation have a long history since computers and digital systems were widely used. At present, researchers have put forward various methods for computer composition, among which the influential ones are hidden Markov chain, rule-based system, music grammar, genetic algorithm, NN technology, etc.

Zheng and Lu used LSTM (long short term memory network) to process blues music of twelve bars and realized the generation of chords and melody in blues music [8]. The hidden layer of the model uses four LSTM modules, the input is the current note, and the output is the predicted note at the next moment. Jenke et al. mainly introduced the related research on algorithmic composition using recursive NN. For the possible gradient vanishing problem, the LSTM algorithm that avoids the gradient vanishing problem is used [9]. Zhang et al. applied generative adversarial networks to algorithmic composition and created the MidNet popular melody generation system [10]. In this network structure, the CNN (convolutional neural network) used by both the generator and the discriminator is trained by converting the midi format data set into a piano roll and inputting it into the network. Then the generator inputs random noise and generates music melody, and then the discriminator will make a true or false judgment on the generated melody. Majumder et al. mainly used the sampling of audio data and mainly designed and innovated the structure of NN [11, 12]. However, this method has certain limitations on the accuracy of preprocessing of music data. Hong et al. adopted a trained LSTM to predict the next note in a monophonic melody and used reinforcement learning to enhance it [13].

With the continuous development of various disciplines, scholars have done a lot of work in the research of music emotion. People gradually recognise people's response mechanism to emotion, establish a unified emotional standard, and establish an open and correct corpus. The unified algorithm evaluation system has continuously promoted the development of emotion recognition technology.

Jiang et al. used the SVM (support vector machine) classification algorithm to extract the spectral features of music and perform sentiment classification [14]. Mattei et al. studied a variety of acoustic features, including low-level features and features such as melody, pitch, and high-level genre, style, etc.; these features were then reduced to a D-dimensional space and associated with semantic features. Finally, automatic recognition of music emotion was done using k-nearest neighbor algorithm [15]. Kaya and Salah explored the effectiveness of random forest classification algorithm in music emotion recognition [16]. Compared with the SVM classification algorithm, this method has greater advantages in generalization and robustness against noise and is very suitable for audio classification tasks. Nordström and Laukka used a continuous emotional mental model and used regression modeling to predict the emotional value of music, using two fuzzy classifiers to measure the emotional intensity to identify the emotional content of music [17]. Yun et al. completed music emotion classification by extracting the pitch, width, and brightness features of music frequency domain [18]. Wang et al. used the SVM method to identify the emotional type of music by extracting the spectral features of music and training these features [19].

The related literature of algorithmic composition and emotion recognition is thoroughly examined in this paper, and a composition and emotion recognition model based on a machine learning algorithm is proposed. According to the information entropy of pitch and intensity, this paper extracts the main melody track. Second, take note features and extract bar features. Finally, the cosine of the vector included angle is used to judge the similarity between feature vectors of several adjacent sections, allowing the music to be divided into multiple segments. The speed, melody direction, intensity, tempo, rhythm change, major third degree, minor third degree, and timbre of each segment are extracted using digital music feature extraction technology, and the emotion of each segment is analyzed using a music emotion model. This paper employs a two-layer filtering mechanism in order to improve retrieval speed. To begin, dissimilar music is quickly filtered out based on time length and category vector. The user is then presented with the most similar music, which is calculated using the exact similarity calculation formula. The study found that the model's retrieval speed is faster, its accuracy is higher, and all indexes are high.

## 3. Methodology

### 3.1. Algorithm and Emotion Recognition

The regular vibration of the vocal body produces music, which is a type of sound art. The composer's inspiration and music creation rules, which primarily include the melody, interval, harmony, chord, mode, and form of music [20], are used to create music. Music's allure stems from the unpredictable nature of creative motivation, and the new auditory experience it provides can often elicit emotional resonance. Music can convey emotions and regulate the mood of listeners as an important part of human life. It is an important aspect of emotional music, and the relationship between computer music, music, and emotion has sparked a lot of research. The various elements of music work together and have a constantly changing expressive force. Melody is the foundation of music, while other elements are the branches and leaves. The image of music will change to varying degrees as each element changes. Melody is a musical sound movement that is organised and harmonious according to certain rules. It is the most common way for musical works to express their feelings. Melody is the heart of music, the foundation of its creation, and the expression of music's image and thought. The pitch relationship between two tones is indicated by the interval. It measures the auditory distance between sounds in degrees, which is a normalised representation method. A sound combination in which multiple tones are arranged according to certain rules is referred to as harmony. The vertical combination of three or more pitches is known as a chord. When it comes to overlapping, it can be done in a third-degree or non-third-degree relationship. The absolute height of a sound is expressed by its phonetic name, which is the expression of its pitch frequency. Every song has a tonic, whose tuning height is represented by key signature and whose height is the key of the scale. Form is a musical structure that combines people's cognition of certain music works in a specific cultural context, and it is a summary of the theoretical laws of music. The smallest unit of sound behaviour in music is the note. A note is a sound that has a specific time length and frequency. In addition, the intensity and timbre of notes should be taken into account when describing them. We can derive the basic characteristics of notes from this: pitch, dynamics, duration, and timbre. Digital music is a new genre of music created with computer technology, stored in digital format, and distributed via digital media technologies like the Internet. Digital music, in comparison to traditional music, has taken on new characteristics as a result of the rapid advancement of digital technology.

The algorithm is a logical and systematic instruction for solving a problem that represents the description of a specific problem and the strategy for solving it. Through normative data input, an excellent algorithm can produce effective and standardized output results in a specified amount of time. Musical elements, writing logic, algorithm, structural model or rule system, and a series of composing techniques formed by matching algorithm thinking with the smallest decision-making model in composition thinking are all examples of algorithm concepts. Computer music differs from traditional music in terms of how it deals with sound, as well as the principles of sound creation and organisation. The creator's perspective and the computer's automatic learning of big data are two common approaches to computer composition. From the perspective of the creator, it is necessary to condense a large number of music-making rules into a single routine. This method produces high-quality music, but it takes a lot of manpower to establish rules and routines in the early stages. Big data [21, 22] automatic learning composition allows computers to learn the laws in music data and then compose music using calculators. Using a computer to learn from big data music can save time and money, and the music generated is more diverse. The way music is processed, manufactured, and organised differs significantly from traditional music. The irrelevance between playing method and timbre breaks through the quantitative limit of timbre [23]. Digital music has various sound effects, and its sound is produced by a point oscillator. However, at this time, the computer is unable to create music that reflects subjective emotion and thought. It is even more difficult to meet people's requirements for pleasant music by simply using a computer to compose music using an algorithm. And, like words, music has emotional connotations. The process of establishing music characteristics and music database is shown in Figure 1.

Music emotion is an essential feature of music, and more research on music information behaviour shows that emotion is an important standard used by people when retrieving music. In fact, there is no such thing as pure musical emotion, and emotion is only meaningful when it is associated with people. When it comes to the same emotion, everyone has different reactions. As a result, if you want to share your musical emotional experience with others, you must express music using a specific rule and symbol, and the same rules and symbols represent the same emotional expression in different types of music. Music emotion recognition, which is one of the important research directions in digital music, is at the heart of emotion-based music retrieval. Computers are unable to perceive the emotions contained in music. As a result, we should summarize the related elements of music into mathematical models and conduct quantitative analysis of them, so that the computer can recognise the emotional connotation of music based on its musical characteristic parameters and rules. Everyone's emotional response to music is a series of brain reactions following the acquisition of characteristic information from the music, with the results reflected in expression and psychological feelings. We must first understand the classification and expression of emotion types in order to study the relationship between music and emotion. Individual needs and desires mediate emotion, which is a psychological state. Emotion is difficult to quantify because it is complex and subjective, and different people have different levels of understanding of it. People have deepened their understanding of emotional types by constantly exploring the changing rules of emotions. At different points in time, a complete piece of music may have emotional changes. Music can be divided into two types of rhythms: fast and slow. Gentle rhythm refers to a slow-changing rhythm. The abrupt rhythm, on the other hand, is a rapidly changing rhythm. Music with a smooth rhythm can evoke a sense of calm, whereas music with an abrupt rhythm can evoke a strong sense of emotion.

### 3.2. Algorithm Composition and Emotion Recognition Model Construction Based on Machine Learning

Based on the deep learning theory [24], aiming at the problems existing in the current algorithmic composition system, this chapter puts forward a new NN structure of music creation from the perspectives of machine learning and music theory creation and constructs a music emotion recognition model. Different music formats have different structural characteristics and extraction methods [3, 25]. This section determines the format of music, making preparations for the extraction of emotional features of music. Generally, music files include three categories: sound files, MIDI files, and module files. MIDI file is a binary file that records the sequence of MIDI instructions. Its basic structure consists of header file and data description. In this paper, MIDI files are selected as experimental objects. The reasons are as follows: ① accurate sampling; ② easy feature extraction; ③ occupying less space; ④ high utilization rate. To begin, obtain the corresponding music score data and music data in MIDI format; after obtaining the music data, it is necessary to create a music data set in accordance with the standard; then, data normalisation, note extraction from music in MIDI format, and other preprocessing operations must be performed on the data input into the network. Multiple audio channels are usually used in MIDI music production because the music is more stereo and beautiful. The main melody is first identified from the MIDI format files in this paper. Input a classical music database in MIDI format, set initial notes to randomly generate music, collect the generated music, and construct a music generation sample database, marked as 0; mark the training data set as 1. Simultaneously, a binary classification model is built to pretrain the CNN network. The music sequence is generated by the LSTM network by setting the initial notes. LSTM, Dropout, Dense, Softmax, and other network layers are commonly used in this paper. After creating the appropriate music generation network, the network must be trained using the appropriate deep learning framework. The specific training scheme is to iteratively optimize it using cyclic operations until a satisfactory result is obtained or the specified number of iterations is reached.  Figure 2 depicts the algorithm's emotion recognition flow.

This model is based on the chess game concept. The generated model is optimized by the Reward function, so that the generated music and the training sample have as much confusion as possible, and the recognition output probability of the classification network CNN is closer to 1; that is, the difference between the generated sample and the training sample cannot be distinguished, and music with similar style and theme to the training sample cannot be distinguished. The music feature analysis model is divided into two sections: one for extracting the main melody and another for extracting the musical emotional features from the main melody and constructing the musical emotional feature vector. The process of NN training is essentially the updating of weights. To update the weight between each neuron, the samples propagate forward through NN to get the output of the output layer and then backward to minimise the difference between the output of the output layer and the sample label. In this paper, a music evaluation function, Reward, is proposed, which can monitor and adjust the generated music in real time, make up for the deficiency of using LSTMNN alone for algorithm composition, make it closer to the composer's creative thinking, and meet the needs of the audience. In most music, the pitch of the main melody is generally higher than that of the accompaniment melody, and the basic contour algorithm is applicable to most music. However, for a small number of music with higher accompaniment melody, we cannot just use the pitch feature as the criterion to judge the main melody, so the basic contour algorithm has limited effect. To solve this problem, this paper proposes an improved contour algorithm based on track features to extract the main melody.

In order to improve the effectiveness of Reward function introduced in this paper, the reference value 1 is subtracted when calculating the probability, as shown in the following formula:

(1) $$\begin{array}{c} p_{\left(\text{CNN}\right)}=\left\{\begin{array}{cc} 0, & \text{fort}<T,\\ D_{\varphi }\left(a_{1:T}\right)-0.5, & \text{fort}=T. \end{array}\right) \end{array}$$

If a piece of music has the interval difference between the adjacent notes in the *a* group greater than the octave, the remaining *b* group is less than or equal to the octave. It can be expressed by the following formula:

(2) $$\begin{array}{c} g_{1}\left(x\right)=\frac{a*0+b*1}{a+b}. \end{array}$$

In order to make the generated music more aesthetic, the following standards are set here:

(3) $$\begin{array}{c} I_{b}\in \left\{0,2,3,4,5\right\},\\ I_{bb}\in \left\{0,2,3,4,5,7\right\},\\ I_{⟶p}\in \left\{6,7,9,10,12\right\},\\ N_{i=1}\in \left\{1,2\right\}. \end{array}$$

Among them, *I*_*b*_, *I*_*bb*_, and *I*_⟶*p*_, respectively, represent the interval sample values corresponding to the measures within the measure, between the measures, and to the climax. *N*_*i*=1_ is the number of minor second intervals in a piece, and the minor second can highlight the tension of the interval. If there are more than four consecutive notes at the same pitch and duration in a piece, this parameter will be recorded as 0; otherwise it will be 1.

(4) $$\begin{array}{c} g_{3}\left(x\right)=\left\{\begin{array}{cc} 1, & \frac{1}{n-1}\left|\sum_{i=1}^{n-1}{\text{interval}}_{i}\leq 4\right|,\\ 0, & \text{else.} \end{array}\right) \end{array}$$

The normalisation strategy in this system adopts the Min-Max scaling method, as follows:

(5) $$\begin{array}{c} X_{\text{normal}}=\frac{X-X_{\min}}{X_{\max}-X_{\min}}, \end{array}$$

where *X*_normal_ represents the normalised value of the digitized note data. *X* represents the digitized note data, *X*_min_ represents the digitized minimum value of note data, and *X*_max_ represents the digitized maximum value of note data.

The algorithm's quality evaluation mechanism plays an important role in improving the quality of music generation in the next step. This paper evaluates the quality of music from both subjective and objective perspectives in order to test the generating effect of algorithmic composition. The learning rate indicates how quickly weights are updated during the training process. The larger the amplitude of updating weights each time, and the faster the initial convergence speed, the higher the learning rate. However, an excessively high learning rate may cause the network to cross the minimum point, making convergence difficult. With the right learning rate, the objective function can converge to the local minimum in a reasonable amount of time. Music emotion recognition is the process of associating music with specific emotions based on the characteristics of the music and given reasoning rules. Emotion recognition is a mathematical mapping process that converts the features of dimensional music into dimensional emotion space. The main melody's relevant features are extracted from the melody of the alternative tracks in this paper to determine the likelihood of each track channel containing the main melody. The higher the score is, the more likely the main melody will be included. Six features of the alternative track melody are extracted based on the musical theory characteristics of the main melody when the related features of the main melody are extracted. These six characteristics are sound source balance, main volume, pronunciation area, loudness area, average pitch, and average sound intensity. Music is a kind of time series. In this paper, LSTM network is used to generate music series. LSTM has a special function of sequential memory. On the basis of ordinary multilayer NN, the structure adds the horizontal connection among the units in the hidden layer. Through a weight matrix, the previous information can be connected to the current task; that is, the next sequence action can be predicted by the previous generated sequence. After the data set is made, the data preprocessing of the data set will be carried out. Its purpose is to make the note data input to NN have a unified standardization standard, thus effectively reducing the number of event types in huge data and effectively improving the generalization ability of the system. It contains many core musical data expressions.

In this paper, we use information entropy to evaluate the amount of information in each track of MIDI file. The formula of entropy is as follows:

(6) $$\begin{array}{c} H\left(p\left(x\right)\right)=-\sum p\left(x\right)\log_{2}^{p\left(x\right)}, \end{array}$$

where *p*(*x*) is the probability density function. The input *s*_*j*_ of each intermediate layer unit is calculated by using the input sample *X*=(*x*_1_, *x*_2_, *x*_3_ …, *x*_*n*_), the connection weight *W*_*ij*_, and the threshold *θ*_*j*_, and then the output *b*_*j*_ of the intermediate layer unit is calculated.

(7) $$\begin{array}{c} s_{j}=\sum_{i=1}^{n}w_{ij}x_{i}-\theta_{j},\;j=1,2,3,\ldots ,p,\\ b_{j}=f\left(s_{j}\right)=\frac{1}{1-e^{-s_{j}}},\;j=1,2,3,\ldots ,p. \end{array}$$

Global error of the calculated network:

(8) $$\begin{array}{c} E=\frac{1}{2}\sum_{i=1}^{q}{\left(y_{i}-c_{i}\right)}^{2}. \end{array}$$

The changing intensity of rhythm can be expressed by the length and intensity of notes in a passage, and the formula is as follows:

(9) $$\begin{array}{c} \text{Rhy}=\sum_{i=1}^{n-1}\left|\frac{I_{i+1}-I_{i}}{D_{i}}\right|. \end{array}$$

The main melody track typically has a large number of notes, and the number of notes in the main melody track should not be less than half of the average number of notes in each track. As a result, before determining the main melody track, tracks with less than half the average number of notes should be eliminated. Musical emotion cannot be expressed solely through the basic information contained in musical notes, and musical emotion analysis must take into account the organisational structure and changing rules of musical notes. As a result, we divide music features into two levels: high-level features and note features, based on the composition form of music features and the audience's hierarchical cognitive process of music features. Following the division of the music into segments with distinct emotions, the forms and methods of music expression are investigated, and some features that have a significant impact on music emotions are chosen to represent music. For each segment, feature extraction is performed, and the extracted features are used to create the segment's feature vector. In this paper, the introduction of attention mechanism will assign different attention sizes to each part of the frame, reflecting the influence degree of each original information on the current information. This number is also the attention size assigned to each word by attention mechanism when learning the current information. When new information is introduced, the training efficiency will be improved.

## 4. Result Analysis and Discussion

This section conducts an experimental comparison of various models in order to verify the performance of the algorithm composition and emotion recognition model based on machine learning proposed in this paper. The network model in this paper is created using Matlab. To begin, create two large loops. After that, the data blocks are then input into the set network model, and the output results are obtained after weight calculation. To ensure the experiment's objectivity, the same training set is used for all algorithms, and the number of network layer units is set to 512 with 200 iterations. Tansig and Logsig are the excitation functions for the network's hidden layer and output layer, respectively. Each note sequence corresponds to a one-hot vector and is 192 characters long.  Table 1 shows the parameter values set by the network in the training process.

The loss value specifies how the difference between the prediction result and the actual label should be calculated. Because note prediction is a multiclassification problem, the categorical cross-entropy function is chosen because of its high performance. The distance between the predicted value and the real value can be minimised by minimising the cross-entropy, achieving the ultimate goal of training. This chapter examines the impact of network parameters on experimental results by looking at the number of iterations. The influence of the number of iterations on the loss value is shown in Figure 3.

The findings show that the longer iteration times are, the more weight parameters are learned and adjusted, which can improve the model's accuracy to some extent. And as the number of iterations increases, the loss function decreases more slowly. When learning and training a NN, the numerical distribution changes dramatically as the number of layers increases, accompanied by error accumulation. The resulting layer-by-layer superposition will drastically alter the high-level input distribution. As a result, the normalisation strategy can be used to process the data distribution to the [0, 1] interval in order to reduce the impact of distribution change. The training set is processed using feature analysis, the emotional feature quantity is used as the model's input, and the classification result is used as the model's output. The error results of different music algorithms are shown in Figure 4.

It can be seen that the error of the music algorithm generated in this paper is the smallest, and its performance is better. In this network, the more units in the hidden layer, the stronger the network's ability to learn abstract data features. The dimension of hidden layer has an important influence on the experimental results, but the more layers there are, the larger the calculation amount of NN will be. Comparison of algorithm recall results is shown in Figure 5.

According to the data analysis in Figure 5, the recall rate of this algorithm is higher than that of the other two algorithms. This algorithm has certain reliability. This chapter verifies the quality of music generation through professional evaluation. 100 music professionals from a university were invited to comprehensively grade 30 samples generated by each model. The results are shown in Table 2.

As can be seen from Table 2, the music generation algorithm in this paper has more advantages in results. This proves the effectiveness of the model in music generation, and it can be seen that the network model constructed in this paper has stronger practical value. In this paper, the emotional classification of music is realized by fusing the time domain features, frequency domain features, auditory spectrogram features, and nonlinear Hurst parameters of music. Through experiments, the accuracy of emotion classification of different algorithms is shown in Figure 6.

It is clear that this model has a higher retrieval accuracy. The results confirm the model proposed in this paper's validity and correctness. In this paper, choose an appropriate training set as the network's input and constantly revise the network's connection weights and thresholds to make it converge. Finally, the emotion recognition model is used to identify the emotion of the music in the test set, and the algorithm's accuracy is evaluated. The emotion recognition accuracy of different algorithms is shown in Figure 7.

When compared to the results of three different algorithms for accurately recognising emotion samples, the algorithm in this paper has a better effect, with higher generalization, stability, recognition rate, and practical value. Several experiments are carried out in this chapter to verify the performance of the algorithm and model proposed in this paper. The model's emotion recognition accuracy is up to 93.78 percent, and the algorithm recall rate is up to 96.3 percent, according to the experimental analysis. The model's retrieval speed is quick, and its accuracy is excellent. Many results show that the recognition method used in this paper is superior to other recognition methods in terms of recognition ability, and the emotion recognition results are reliable.

## 5. Conclusions

Research on an efficient music generation algorithm and emotion recognition model has become a research hotspot as artificial intelligence technology matures. The construction of an emotion recognition model of composition is a multidisciplinary research topic. This paper builds an algorithm composition and emotion recognition model based on an in-depth study of machine learning. This paper examines the workflow of a music emotion recognition system and summarizes the contents of digital music emotion recognition and music features. The features are used to represent music, and then algorithms are used to analyze the features to determine the emotional categories of music. The model's emotion recognition accuracy is up to 93.78 percent, and the algorithm recall rate is up to 96.3 percent, according to the experimental analysis. The segmented emotion recognition method proposed in this paper can better show the movement of music than the whole music emotion recognition method. It has a strong ability to recognise emotions. The experimental results show that this recognition method has superior recognition ability, fast retrieval speed, and certain reliability when compared to other recognition methods. The method proposed in this paper is feasible and effective, and it produced the expected outcomes. On the level of computer-aided music creation, artificial intelligence music is expected to help creators fill the thinking gap in creation in the future, and users will be able to choose the most appropriate candidate sequence to increase creator inspiration. You can also recreate entirely new music in the style of specific musicians and composers. This study, however, has some flaws due to the influence of our knowledge level and time constraints. We can continue to research the emotional model in order to more scientifically represent the emotional categories of music in future work.

## Figures and Tables

**Figure 1:** Emotional characteristics of music and the establishment process of music database.

**Figure 2:** The algorithm emotion recognition flow in this paper.

**Figure 3:** Influence of iteration times on loss value.

**Figure 4:** Generate error results of different music algorithms.

**Figure 5:** Comparison of algorithm recall results.

**Figure 6:** Comparison of accuracy of different algorithms in emotion classification.

**Figure 7:** Different accuracy of emotion recognition algorithm.

**Table 1:** Parameter values of network settings in this paper.

Serial number	Parameter	Set value
1	Input layer-neuron	9
2	Hidden layer-neuron	20
3	Output layer-neuron	7
4	Epochs	200
5	Batch_ size	64
6	Loss	Categorical_crossentropy
7	Optimizer	Rmsprop
8	Save_ number	20
9	Activation	Softmax activation function

**Table 2:** Evaluation of music generation quality.

Model	Melody	Rhythm	Harmony	Expressive force	Satisfaction (%)
HMM model	6.36	7.15	6.47	6.18	65.03
MCMM model	7.59	7.34	8.01	7.03	69.34
Seq GAN model	6.28	6.84	7.78	6.35	63.17
RL-RNN model	6.54	6.58	6.97	5.84	59.93
RFCM model	5.89	5.13	6.74	6.62	58.46
Model of this paper	7.76	7.45	8.03	7.16	74.89

## Data Availability

The data used to support the findings of this study are available from the corresponding author upon request.
